# The biological functions and related signaling pathways of SPON2

**DOI:** 10.3389/fonc.2023.1323744

**Published:** 2024-01-09

**Authors:** Jingrun Zhang, Ge Liu, Yuchen Liu, Pei Yang, Junyuan Xie, Xiaowei Wei

**Affiliations:** ^1^Zhongshan Clinical College, Dalian University, Dalian, China; ^2^Laboratory of Orthopedics, Affiliated Zhongshan Hospital of Dalian University, Dalian, China; ^3^Department of Neurology, The Third Affiliated Hospital of Xinxiang Medical University, Xinxiang, China; ^4^Department of Breast Surgery, The First Affiliated Hospital of Zhengzhou University, Zhengzhou, China

**Keywords:** SPON2, biomarker, biological function, signaling pathway, WNT/β-catenin

## Abstract

Spondin-2 (SPON2), also referred to as M-spondin or DIL-1, is a member of the extracellular matrix protein family known as Mindin-F-spondin (FS). SPON2 can be used as a broad-spectrum tumor marker for more than a dozen tumors, mainly prostate cancer. Meanwhile, SPON2 is also a potential biomarker for the diagnosis of certain non-tumor diseases. Additionally, SPON2 plays a pivotal role in regulating tumor metastasis and progression. In normal tissues, SPON2 has a variety of biological functions represented by promoting growth and development and cell proliferation. This paper presents a comprehensive overview of the regulatory mechanisms, diagnostic potential as a broad-spectrum biomarker, diverse biological functions, involvement in various signaling pathways, and clinical applications of SPON2.

## 1 Introduction

Spondin-2 (SPON2), also referred to as M-spondin or DIL-1, is a member of the extracellular matrix (ECM) protein family known as Mindin-F-spondin (FS) (1). The SPON2 protein, consisting of 243 amino acids (2), is a secreted ligand that interacts with leucine-rich repeat-containing G protein-coupled receptors to enhance the WNT signaling (3). The expression of SPON2 can be regulated by hormones or epigenetically. SPON2 expression is induced by the thyroid hormone (4, 5) in human cancer. Kim JW et al. observed a negative correlation between the methylation status of SPON2 and its gene expression (6). Furthermore, the expression of SPON2 is associated with microRNAs (miRNAs) (7).

As widely acknowledged, SPON2 has emerged as a broad-spectrum biomarker. In recent years, reports of up-regulation of SPON2 in various tumor types have proliferated. The serum index of SPON2 is highly sensitive to tumor diagnosis, according to research findings (8, 9). For some non-tumor diseases, the change of SPON2 expression also has important potential significance for the diagnosis of the diseases.

The multifaceted biological functions of SPON2 have been extensively documented. Notably, research studies have elucidated the pivotal regulatory role played by SPON2 in tumor progression and metastasis. For example, SPON2 promotes the proliferation, migration, and invasion of stomach cancer (STAD) cells in STAD (10). SPON2 also plays a pivotal role in tissue morphogenesis and regulation of cellular proliferation in physiological contexts. Yamada W et al. emphasize its indispensable contribution to midfacial, limb, and lung morphogenesis during embryogenesis (3). Concurrently, SPON2 functions as a regulator of the host’s innate immune response by facilitating the recruitment of inflammatory cells and activation of the intrinsic immune system (11).

SPON2 exerts diverse biological functions by participating in multiple signaling pathways. It has been documented that SPON2 exhibits simultaneous binding affinity towards LGR4, LGR5, and LGR6 receptors, thereby enhancing the canonical WNT signaling pathway (12, 13). The activation of the NF-κB pathway by SPON2 plays a crucial role in promoting osseous metastasis in lung adenocarcinoma (LUAD) (14). SPON2 promotes the proliferation and metastasis of ovarian cancer (OV) by activating the FAK/SRC signaling cascades (15). The upregulation of SPON2 enhances the activation of the Notch signaling pathway, thereby contributing to the progression of STAD (16). Jin YR et al. discovered that SPON2 exerts a crucial regulatory role in the morphogenesis of midface, limb, and lung during development by modulating the WNT/β-catenin signaling pathway (17, 18). Furthermore, SPON2 has the potential to function as a positive regulator of bone metabolism through the activation of the canonical WNT/β-catenin signaling pathway (19).

Because of the specific expression of SPON2 in tumor tissues, it makes SPON2 an ideal target for researchers to develop targeted therapy and immunotherapies for tumors. Currently, there have been notable advancements in the clinical application of SPON2. For example, in ampulla adenocarcinoma, SPON2 RNA fusion could be a potential target for therapy (20). In metastatic colorectal cancer, targeting SPON2 helps overcome resistance to anti-angiogenic therapies (21). In prostate cancer, SPON2 can be used as an antibody-based radiotherapy target (22). The aforementioned points will be expounded upon in the subsequent sections.

## 2 Regulation of SPON2 expression

SPON2 is an ECM-attached protein. The SPON2 gene is transcribed and translated, converting the genetic information encoded by the gene into proteins, which then combine with the ECM to play a role (23). The expression of SPON2 can be modulated by hormonal factors or epigenetic regulation. The expression of SPON2 is induced by thyroid hormone (4, 5) in human cancer. Hypomethylation of the SPON2 promoter results in an upregulation of SPON2 expression in prostate cancer and meningioma (6). Conversely, the presence of middle or high methylation levels in the SPON2 promoter leads to diminished expression of SPON2, which exhibits a strong association with favorable outcomes among patients diagnosed with acute lymphoblastic leukemia (24). These observations suggest that the expression of the cancer-associated SPON2 gene is regulated at the transcriptional level, thereby implying its potential as a prognostic marker in cancer patients (11).

MicroRNAs (miRNAs), consisting of 20-22 nucleotides, represent prominent examples of small RNAs. They specifically bind to the 30 untranslated regions (30utr) of target mRNA molecules and exert regulatory control over gene expression by impeding translation or inducing mRNA cleavage, thereby repressing protein synthesis. SPON2 plays a crucial role in the activation of the WNT/β-catenin signaling pathway, regulating various pivotal processes associated with tumor progression, including tumorigenesis, cell proliferation, migration, and invasion. Xu Y et al. also demonstrated that miR-493 exerts inhibitory effects on liver cancer development by suppressing the expression of SPON2, thereby attenuating the WNT signaling pathway (25). In their study, Kun Chen et al. demonstrated that miR-497-5p effectively suppressed the expression of SPON2 in glioblastoma (GBM) tumors, thereby inhibiting the WNT/β-catenin signaling pathway and subsequently reducing cellular metastasis (7). Furthermore, Kang et al. demonstrated a significant correlation between Notch signal transduction and SPON2 expression through cDNA microarrays and *in vitro* studies (16). A comprehensive understanding of the upstream and downstream regulatory factors of SPON2 could provide valuable insights for anti-tumor therapy targeting molecular markers. We summarize the relevant regulatory mechanisms of SPON2 in **Figure 1**.

**Figure 1:** The regulatory mechanisms of SPON2. The expression of SPON2 is regulated by the Notch signaling pathway and thyroid hormone, while miRNA inhibits translation or induces cleavage of SPON2 mRNA. Furthermore, the SPON2 protein participates in related signaling pathways to modulate biological functions, such as the PI3K/AKT/mTOR signaling pathway and the FAK/SRC signaling pathway.

## 3 SPON2 as a broad-spectrum biomarker in different diseases

### 3.1 SPON2 as a broad-spectrum biomarker for tumors

In recent years, there has been a growing body of literature highlighting SPON2 as a promising biomarker. Elevated levels of SPON2 have been observed in the serum and tumor microenvironment of patients with multiple tumors. Furthermore, it has gained widespread recognition as a reliable biomarker for prostate cancer (PRAD) and ovarian cancer (OV) in clinical settings (11). The upregulation of SPON2 in various tumors was demonstrated in **Figure 2**.

**Figure 2:** The expression of SPON2 in various cancer types. The figure illustrates various cancer types through different colors. KIRC, kidney clear cell carcinoma; LSCC, laryngeal squamous cell carcinoma.

#### 3.1.1 Urinary system tumors

Romanuik TL et al. observed a significant upregulation in the expression of both mRNA and protein levels of SPON2 in prostate cancer (PRAD) (26). Parra-Cabrera C et al. identified prostate-specific antigen (PSA) and SPON2 present in the bloodstream as potential combined screening tools for diagnosing PRAD (27). Qian XL et al. conducted a comparative study involving 13 healthy elderly men and 70 patients with prostate cancer, revealing that the optimal critical value of SPON2 for achieving the highest sensitivity (100%) and specificity (84.6%) was determined to be 8 μg/L. Furthermore, the positive predictive value was calculated as 97.2%, while the negative predictive value remained at a robust 100% (28). The study conducted by HU BP et al. involved the treatment of 85 patients diagnosed with prostate cancer. These patients were categorized into two groups based on the presence or absence of bone metastasis, namely the bone metastasis group (43 cases) and the non-bone metastasis group (42 cases). Following statistical analysis, a threshold value of 8 μg/L for SPON2 was identified as a positive indicator, exhibiting a sensitivity of 86.05% and specificity of 83.74%. This research contributes novel diagnostic insights for PRAD bone metastasis (29). Lucarelli G et al. analyzed serum samples from 286 prostate cancer patients and 68 individuals without malignant tumors, demonstrating that SPON2 exhibited superior predictive value compared to serum sarcosine, free PSA percentage ratio, and total PSA. These findings suggest that SPON2 has the potential to significantly enhance PRAD detection accuracy (8). Although the tissue sources and patient populations differ among the aforementioned studies, Qian XL and HU BP et al. concur that SPON2>8 μg/L holds significant value in PRAD detection. This implies that SPON2 can replicate this phenomenon across diverse populations, thereby endorsing its utility as a clinical detection indicator for enhanced stability and reliability.

The overexpression of SPON2 is closely associated with kidney clear cell carcinoma (KIRC) and bladder cancer (BLCA). Zhao X et al. identified differentially expressed genes (DEGs) in 165 patients with BLCA based on the TCGA database and evaluated the association between immune/interstitial scores, clinical features, and prognosis. They observed a significant correlation between SPON2 expression and bladder cancer prognosis, suggesting its potential as a prognostic biomarker for BLCA (30). Using expression data from TCGA and GEO databases, Ma HM et al. assessed the SPON2 expression in KIRC and observed a significant overexpression of SPON2 in 94 cases of KIRC. Furthermore, they found a significant correlation between SPON2 expression and tumor stage, Fuhrman grade, as well as postoperative recurrence in patients with localized lesions. These findings suggest that elevated levels of SPON2 could serve as a valuable prognostic biomarker for patients with localized KIRC (31).

#### 3.1.2 Digestive system tumors

The overexpression of SPON2 can serve as an independent prognostic indicator for colorectal cancer (CRC), stomach cancer (STAD), and liver cancer (LIHC). Zhang Q et al. observed an upregulation of SPON2 mRNA expression in 180 cases of CRC compared to adenomas. Furthermore, this increase in SPON2 mRNA expression exhibited a significant correlation with the pathological stage of CRC patients. Notably, plasma SPON2 demonstrated a sensitivity and specificity of 100% and 90%, respectively, at a concentration of 12.1μg/L. These findings suggest that SPON2 exhibits comparable or superior performance in CRC when compared to prostate cancer as a diagnostic marker. Additionally, plasma levels of SPON2 were found to be upregulated in CRC and decreased postoperatively, indicating its potential as an independent diagnostic and prognostic biomarker for CRC (11). A total of 64 samples of CRC tissues and adjacent tissues were collected by Liu H et al., and the mRNA and protein expression levels of SPON2 in these tissues were assessed using qRT-PCR and immunohistochemistry. The results revealed a significant increase in both mRNA and protein expression levels of SPON2 in CRC tissues compared to adjacent tissues. Furthermore, the expression levels of SPON2 in CRC tissues were higher than those observed in normal tissues, although statistical significance was not reached when compared with adjacent tissues. However, it is worth noting that the sample size for this study was limited, thus necessitating further large-scale investigations (32). Metastasis-associated colon cancer 1 (MACC1) plays a crucial role in promoting the metastasis of colon cancer. Through an extensive genome-wide analysis of gene expression, researchers have successfully identified SPON2 as one of the pivotal downstream effectors regulated by MACC1. Furthermore, they propose that SPON2 could serve as an independent prognostic indicator for CRC metastasis and overall survival without disease recurrence (9). Based on the analysis of 60 paraffin-embedded biopsy samples, encompassing patients with colorectal adenoma (CRA), malignant polyps, and CRC, Žlajpah M et al. observed a proportional increase in SPON2 expression corresponding to the tumor’s malignancy (33).

Lu HM et al. identified SPON2 as an oncogene in STAD progression (10). Rajkumar T et al. investigated plasma protein levels in 58 patients with STAD and 18 patients with normal/non-malignant gastric disease, revealing differential expression of SPON2 in STAD. These findings suggest that SPON2 may serve as a promising diagnostic marker and therapeutic target for STAD; however, the limited sample size warrants further investigation (34). The study conducted by Jin C et al. involved the analysis of 174 STAD samples using univariate and multivariate methods, leading to the conclusion that SPON2 could serve as an independent prognostic factor for both relapse-free survival and overall survival (35). Kuramitsu S et al. utilized STAD datasets to conduct clinicopathological and prognostic analyses of SPON2 mRNA expression. Immunohistochemistry was employed to evaluate the localization of SPON2 expression, revealing that cancer-associated fibroblast-derived SPON2 may enhance the motility of STAD cells, thereby promoting peritoneal dissemination (PD). These findings suggest that SPON2 could serve as a predictive marker for PD in STAD (36). The aforementioned studies have consistently demonstrated the significant role of SPON2 in STAD diagnosis; however, its specific prognostic value in predicting STAD progression remains unexplored. Furthermore, Feng Y et al. conducted immunohistochemical staining and utilized tissue microarray to assess the expression of SPON2 protein in 107 matched pairs of LIHC and normal liver tissues. The findings revealed that the level of SPON2 protein expression in tumor tissues from LIHC patients could serve as a valuable prognostic indicator for LIHC (37).

#### 3.1.3 Respiratory system tumors

Overexpression of SPON2 has also been associated with lung adenocarcinoma (LUAD), and laryngeal squamous cell carcinoma (LSCC). Manda R et al. demonstrated differential mRNA expression profiles among three small cell lung cancer (SCLC) cell lines, six non-small cell lung cancer (NSCLC) cell lines, and three normal lung tissues. Additionally, they identified genes that were differentially expressed between lung cancer cells and normal lung tissues, as well as between SCLC cells and NSCLC cells. Notably, distinct expression levels of SPON2 were observed between malignant and non-malignant lung cells. However, the study was limited to cellular investigations without further exploration of clinical samples from patients with lung cancer (38). Yuan XP et al. conducted a tissue microarray immunohistochemical analysis (TMA-IHC) to examine the expression of SPON2 protein in 280 lung cancer patients, revealing that elevated levels of SPON2 protein were significantly associated with differentiation, positive lymph node metastasis, increased serum carcinoembryonic antigen levels, and poor overall survival. The overexpression of SPON2 protein can serve as an independent prognostic biomarker for lung cancer patients (39). Chen ZP et al. reported an upregulation of SPON2 expression in LUAD patients, suggesting that targeting SPON2 in the tumor microenvironment could enhance the efficacy of LUAD treatment. However, this study only analyzed T1 stage samples from TCGA for LUAD. A comprehensive analysis of changes in SPON2 expression across all stages of lung cancer would provide a more robust diagnostic foundation for the diagnosis and treatment of this disease (40).

Ni HS et al. collected a total of 111 paraffin-embedded LSCC specimens along with adjacent non-tumor tissues, as well as 15 pairs of fresh tissues from patients diagnosed with LSCC. Their findings revealed a significant increase in SPON2 levels within the LSCC tissues compared to the adjacent normal tissues. Furthermore, they observed that elevated SPON2 levels were closely associated with lymph node metastasis, pathological grade, and clinical stage among LSCC patients. The analysis demonstrated that patients exhibiting high expression of SPON2 had a lower overall survival rate when compared to those with low expression levels. These results suggest that SPON2 holds promise as both a novel therapeutic target and prognostic biomarker for individuals affected by LSCC (41).

#### 3.1.4 Genital system tumors

Simon I et al. conducted an ELISA analysis on SPON2 levels in 108 control samples of ovarian cancer (OV) and serum samples from 20 healthy women. The findings suggest that SPON2 holds promise as a novel marker for OV, with the potential to enhance early cancer detection when combined with conventional diagnostic tests (42). Oikonomopoulou K et al. collected serum biochemical parameters from 98 patients with OV before and during chemotherapy. In the univariate analysis, SPON2 was found to have potential implications in predicting chemotherapy response, overall survival, short-term (1-year) survival, progression-free survival, and time to progression (TTP) in patients with OV following chemotherapy (43). In two separate studies targeting distinct populations, Simon I and Oikonomopoulou K et al. reported consistent diagnostic and prognostic value of SPON2 in OV, indicating the reproducibility of SPON2 detection across diverse populations. Zhang LL et al. conducted a comprehensive analysis of SPON2 expression in the sera of 147 cervical cancer (CESC) patients, 92 individuals with benign uterine lesions, and 86 healthy controls. The results showed that the level of SPON2 expression was significantly higher in the cervical cancer group compared to both control groups. Furthermore, after a three-year follow-up period, patients with high levels of serum SPON2 had significantly shorter progression-free survival and overall survival rates than those with low levels of serum SPON2. These findings suggest that increased serum SPON2 expression is associated with tumor invasion, anti-tumor immune response, and overall prognosis in cervical cancer patients. This large-scale study not only included case-control analyses but also long-term follow-up data which has important implications for clinical practice (44).

#### 3.1.5 Other system tumors

Sun R et al. demonstrated that SPON2 functions as an autocrine antagonist of BMP proteins in acute myeloid leukemia, thereby promoting cancer cell self-renewal. Moreover, the expression of SPON2 can serve as a potential tumor marker for predicting unfavorable prognosis in this disease. However, it is worth noting that this study was limited to cellular and animal models, without further investigation on clinical tissue samples (45). Hu XY et al. utilized immunohistochemistry to detect the expression of SPON2 in 12 paraffin specimens of Triple-negative breast cancer (TNBC), corresponding normal specimens adjacent to TNBC, and 20 cases of breast fibroadenoma. The protein expression level of SPON2 was higher in TNBC tissues compared to normal tissues. Analysis from the GEO database revealed that the mRNA expression level of SPON2 was also higher in TNBC than in non-TNBC. These findings suggest that the upregulation of SPON2 is associated with poorer patient outcomes in TNBC. Furthermore, knockdown experiments demonstrated that inhibition of SPON2 significantly suppressed cell proliferation, migration, invasion, and tumorigenesis while promoting apoptosis in TNBC cells. Therefore, these results indicate that SPON2 could serve as a valuable biomarker for diagnosis and prognosis as well as a potential therapeutic target for this subtype of breast cancer. Although detailed studies on the molecular mechanism and protein expression were conducted, it should be noted that further research with larger sample sizes across different populations is necessary to ensure the reliability and generalizability of these conclusions (46).

### 3.2 SPON2 as a broad-spectrum biomarker for non-tumor diseases

SPON2 can serve as a potential biomarker for bronchial asthma (BA), diabetic nephropathy (DN), and ossification of the posterior longitudinal ligament of the spine (OPLL). Zhou P et al. conducted a study analyzing peripheral blood samples from 137 children with BA and 59 healthy children, recording their clinical information, indexes, and pulmonary ventilation function. The findings revealed a significant upregulation of SPON2 in the pediatric BA group compared to the healthy control group. Furthermore, there was a positive correlation between the relative level of SPON2 and the severity of bronchial asthma. Thus, SPON2 is considered an important biomarker for diagnosing and assessing the severity of bronchial asthma (47). Murakoshi M et al. employed real-time fluorescent quantitative PCR, western blot analysis, and immunohistochemical staining to detect SPON2 expression in mouse and human glomeruli, cultured podocellular cells, and urine samples. Their findings revealed elevated levels of urinary SPON2 in patients with type 2 diabetes compared to healthy individuals, suggesting its potential as an early biomarker for monitoring the progression of DN (48, 49). Nakajima M et al. identified SPON2 as a susceptibility gene associated with OPLL (50).

## 4 Biological functions of SPON2

### 4.1 The regulatory role of SPON2 in tumor tissues and its related signaling pathways

Biological function of SPON2 in tumors: SPON2 exhibits diverse effects across different tumor tissues, acting as an oncogene in most tumors, while also acting as a tumor suppressor gene in liver cancer (LIHC) and colorectal cancer (CRC), thereby exerting inhibitory influence on tumor progression. A comprehensive summary of the biological role of SPON2 in tumors and its associated signaling pathways is provided in **Table 1**. Subsequent sections will elaborate on these aspects.

**Table 1:** Summary of the mechanism of SPON2 in the biological function of tumors.

Cell or tissue	Biological function	Signaling pathways	Reference
OV	promotes the growth and metastasis of OV	FAK/SRC signaling pathway	(15)
STAD	promotes tumor progression in STAD	Notch signaling pathway	(16)
STAD	Promotes the proliferation, migration, and invasion of STAD cells	ERK1/2 signaling pathway	(10)
STAD	enhances cell invasion and migration in human STAD	WNT/β-catenin signaling pathway	(51)
LUAD	promotes bone metastasis	NF-κBsignaling pathway	(14)
BRCA	enhances bone metastasis	SPON2/RANKL/LGR4 signaling pathway	(52)
GBM	maintains stem cell traits in GBM	WNT3a/β-catenin signaling pathway	(53)
Schwann cell	drives human Schwann cell transformation, progression, and tumor maintenance	WNT/β-catenin signaling pathway	(54)
LIHC	promotes LIHC formation *in vivo* and *in vitro*	Hippo/Yap signaling pathway	(55)
LIHC	suppresses the progression of LIHC	MAPK signaling pathway	(56)
LIHC	promotes proliferation and migration in human LIHC	WNT/β-catenin signaling pathway	(57)
CRC	suppresses CRC metastasis	WNT5a/FZD7 signaling pathway	(58)

#### 4.1.1 SPON2 as an oncogene promotes tumor metastasis and progression

SPON2 facilitates the metastasis of diverse tumors, which is closely associated with epithelial-mesenchymal transition (EMT). EMT is a pivotal biological process wherein epithelial cells undergo a specific procedure to acquire a mesenchymal phenotype. This transformation empowers malignant tumor cells derived from epithelial tissue to gain migratory and invasive capabilities. SPON2 promotes EMT in various tumors through relevant signaling pathways, thereby fostering the metastatic potential of malignant tumor cells (**Figure 3**).

**Figure 3:** SPON2 facilitates EMT in various tumors by modulating relevant signaling pathways to promote metastasis of tumor cells. EMT, epithelial-mesenchymal transition; STAD, stomach cancer; BRCA, breast cancer; GBM, glioblastoma; TSCC, tongue squamous cell carcinoma; and LUAD, lung adenocarcinoma.

Pan R et al. have demonstrated that SPON2 exerts a promotive effect on the growth and metastasis of ovarian cancer through activation of the FAK/SRC signaling cascade (15). Zhang HB et al. observed a significant up-regulation of SPON2 in STAD specimens and cell lines, which was strongly associated with tumor metastasis. Their study demonstrated that SPON2 facilitates the epithelial-mesenchymal transition (EMT) of STAD cells through activation of the ERK1/2 and WNT/β-catenin signaling pathways (10, 51). Kang HG et al. reported an up-regulation of SPON2 expression levels in both STAD cell lines and patient tissues. Their findings from cDNA microarray and *in vitro* studies demonstrated a significant correlation between Notch signal transduction and SPON2 expression, with the Notch signal promoting cell proliferation, migration, and invasion through increased SPON2 expression (16). The expression and secretion of SPON2 in cancer-associated fibroblasts (CAFs) within STAD tissues have been identified by several scholars. A wealth of evidence suggests that SPON2 expression triggers actin cytoskeletal remodeling, including the formation of prosthetic feet, which is a crucial process for tumor cell motility. Furthermore, SPON2 promotes peritoneal dissemination (PD) by enhancing the motility of STAD cells. However, the regulatory mechanisms governing SPON2 expression in CAFs remain unclear. Further investigation into the factors modulating SPON2 expression in CAFs may provide valuable insights into the intricate relationship between SPON2 and PD (36).

Several researchers posit that SPON2 plays a pivotal role in the promotion of bone metastasis. For instance, Wu M et al. demonstrated that SPON2 augmented migration, invasion, and EMT of lung adenocarcinoma (LUAD) cells *in vitro*, while silencing SPON2 significantly impeded LUAD cell-mediated bone metastasis *in vivo*. Mechanistic investigations have revealed that SPON2 facilitates the migration and invasion of LUAD cells through activation of the NF-κB pathway (14). Yue ZY et al. demonstrated that the interaction between SPON2 and its receptor LGR4, in conjunction with RANKL, facilitates the formation of osteoclastic premetastatic niches, thereby enhancing BRCA bone metastasis (52). Na+/H+ exchange regulatory factor (NHERF-1) is a scaffold protein implicated in tumor regulation and osteogenesis. Alvarez-Carrion L et al. discovered that SPON2 promotes prostate cancer progression by downregulating NHERF-1, thereby enhancing tumor cell migration and proliferation (59).

The study conducted by Kang YE et al. retrospectively examined 214 patients with thyroid cancer and revealed a significantly elevated expression level of SPON2 in thyroid cancer tissues compared to the normal control group. Furthermore, it was demonstrated that up-regulation of the SPON2/GPR48/LGR4 pathway plays a crucial role in promoting tumor aggressiveness in thyroid cancer through the facilitation of ERK phosphorylation. However, it is important to note that this study only tested three cell lines at the cellular level and did not include any animal experiments. Therefore, further investigations using different cell lines and animal models are warranted to validate these findings (60). Zhang LP et al. detected the expression of SPON2 in TSCC specimens and evaluated its correlation with clinical outcomes. The levels of SPON2 were significantly elevated in tongue squamous cell carcinoma specimens, which strongly correlated with lymph node metastasis, clinical stage, and survival in patients with TSCC. These findings from clinical investigations suggest that SPON2 is closely associated with tumor metastasis and has high potential for guiding clinical work (61). Chen K et al. demonstrated that SPON2 facilitates GBM cellular metastasis by activating the WNT/β-catenin signaling pathway (7). Additionally, Liu S et al. demonstrated that SPON2 exerts a potent stimulatory effect on the WNT/β-catenin signaling pathway in glioblastoma (GBM) cell lines. Furthermore, when combined with WNT3a, SPON2 effectively induces the expression of pluripotent stem cell markers. Notably, SPON2 plays a crucial role in promoting self-renewal and inhibiting differentiation induced by retinoid or growth factor deprivation, thereby contributing to the maintenance of stem cell characteristics in GBM (53).

#### 4.1.2 The regulatory role of SPON2 in liver cancer and colorectal cancer

The WNT signaling pathway, as well as the Hippo/Yes-associated protein (Yap) pathway, has been implicated in many human cancers (62). Conboy CB et al. conducted a comprehensive analysis of gene expression data from 200 liver tumors and 50 normal liver samples obtained from the TCGA dataset, revealing significant overexpression of SPON2 in liver cancer (LIHC) as a whole. Furthermore, in a mouse model of LIHC, they observed upregulation of SPON2 along with activation of the WNT/β-catenin and Hippo/Yap signaling pathways, leading to hepatomegaly, enhanced tumor formation, and accelerated progression of LIHC (55). However, contrary research findings have been reported by Zheng C et al., who conducted immunohistochemical tests on 50 pairs of LIHC and corresponding non-tumor liver (CNL) tissues from the Department of Liver Surgery of Nanjing Gulou Hospital and the Affiliated Hospital of Nanjing University School of Medicine. They analyzed the expression level of SPON2 in LIHC tissues and found a low expression level that correlated with poor prognosis. Human mRNA microarray analysis was used to screen for differentially expressed mRNA between overexpressed SPON2 and control LIHC cells. Gene microarray and Western blot analysis revealed significant changes in the MAPK signaling pathway after transfection. Furthermore, *in vivo* experiments demonstrated that SPON2 knockdown increased tumorigenicity in mice following subcutaneous implantation. These findings suggest that SPON2 may function as a novel tumor suppressor gene, inhibiting proliferation and invasion of LIHC through the MAPK signaling pathway (56). ZhangYL et al. conducted gene expression analysis and immunohistochemical detection on 202 pairs of tumor tissues and adjacent non-tumor liver tissues from Renji Hospital affiliated with Shanghai Jiao Tong University School of Medicine, revealing that SPON2 was overexpressed in 52% of LIHC patients. Subsequently, the relationship between SPON2 expression and various pathological parameters was analyzed in 202 LIHC patients, demonstrating that high SPON2 expression correlated with improved overall survival and relapse-free survival compared to low expression. Furthermore, except for SMMC-7721 and HepG2 cell lines, most LIHC cell lines exhibited higher levels of SPON2 expression when compared to human liver THLE-2 immortal cells. This report utilized a large sample size study with clinical relevance analysis, providing stronger evidence than cell or animal experiments and offering valuable guidance for clinical practice (63). According to the aforementioned reports, there exist disparities in both the tissue sample source area and cell line selection between Conboy CB et al.’s study and Zhang YL et al.’s study. Variations in SPON2 expression among different populations and cell lines within LIHC tissues imply distinct effects of SPON2 on LIHC across diverse populations.

The biological role of SPON2 in CRC remains a subject of controversy. Huang CM et al. conducted immunohistochemical double staining analysis on 67 paraffin-embedded CRC tissue specimens from Guangzhou Nanfang Hospital and observed a positive correlation between SPON2 expression, M2-TAM infiltration, and the progression of CRC. Furthermore, through *in vitro* migration assay, transendothelial migration assay (iTEM), and cell adhesion assay, it was discovered that SPON2-driven infiltration of M2 tumor-associated macrophages (TAMs) plays a crucial role in the growth and metastasis of CRC (64). However, Cheng XS et al. established a mouse homologous CRC cell line and developed a lentivirus-based overexpression and SPON2-knockdown mouse model of colitis-associated colorectal cancer (CAC). Their findings demonstrate that SPON2 overexpression significantly suppresses tumor growth *in vivo*, suggesting its direct role as a tumor suppressor in the progression of CRC (65). Dong XM et al. also demonstrated that SPON2 exerts inhibitory effects on the migration, invasion, and metastasis of CRC cells by impeding the interaction between WNT5a and Fzd7 receptor, thereby antagonizing the non-classical WNT pathway mediated by WNT5a/FZD7 in advanced CRC (58). Wu CJ et al. reported a significant down-regulation of SPON2 transcription levels and protein in 85% (68 out of 80) primary CRC tumors from the First Affiliated Hospital of Wenzhou Medical University. While SPON2 was expressed in normal colorectal epithelium, its expression was significantly low or undetectable in 9 CRC cell lines. Notably, overexpression of SPON2 in LS174T and DLD1 CRC cell lines demonstrated an inhibitory effect on cell proliferation, whereas removal of SPON2 using short interfering RNA (siRNA) led to a significant enhancement in cell proliferation for both cell lines. These findings suggest that deficiency of SPON2 promotes tumor growth, while its overexpression can suppress the proliferation and tumorigenicity of CRC cells (66). According to the aforementioned report, variations in cell lines selected for the conducted experiments may account for the inconsistent results. Furthermore, it is worth noting that Huang CM et al.’s study primarily focused on clinical samples from Guangzhou, a coastal city in southeast China, while Wu CJ et al.’s study mainly concentrated on clinical samples from Wenzhou, Zhejiang province. Previous research by Jing F et al. has indicated that disparities in regions, lifestyles (67), and ethnicities (68) can potentially lead to divergent amino acid sequences of SPON2 and subsequently influence its impact on CRC development and progression.

### 4.2 The regulatory role of SPON2 in non-tumor tissues and its related signaling pathways

SPON2 not only facilitates growth, development, and angiogenesis in non-tumor tissues but also plays a pivotal role in inflammation promotion, blood gas barrier maintenance, and liver lipid metabolism regulation. Further elucidation of SPON2’s involvement in various signaling pathways and its implications in non-tumor tissues are comprehensively summarized in **Table 2**. These aspects will be discussed extensively below.

**Table 2:** Summary of relevant mechanisms of SPON2 in the biological functions of physiological processes.

Cell or tissue	Biological function	Signaling pathway	Reference
Osteoblast	boosts osteogenic factor levels in osteoblasts	PI3K/AKT/mTOR signaling pathway	(69)
Osteoblast	promotes osteoblast maturation and mineralization	WNT11/β-catenin signaling pathway	(70)
AER	maintains apical ectodermal ridge	WNT/β-catenin signaling pathway	(71)
Mouse face	regulates facial morphogenesis in mice	WNT9b/β-catenin signaling pathway	(17)
Craniofacial bone	regulates craniofacial patterning and morphogenesis	WNT/β-catenin signaling pathway	(72)
C57MG mouse mammary epithelial cells	regulates novel target genes	WNT3a signaling pathway	(73)
Oocyte-granulosa cells	drives the maturation of the ovarian follicles	WNT/CTNNB1 signaling pathway	(74)
Human pluripotent stem cells	promotes hematopoietic development	WNT/TGF-β signaling pathway	(75)
Lung stem/progenitor cells	controls the expansion and differentiation	WNT/β-catenin signaling pathway	(76)
Human dental pulp stem/progenitor cells	promotes the proliferation and odontogenic differentiation	WNT/β-catenin signaling pathway	(77)
LEC	inhibits lymphangiogenesis and downstream impairment	AKT/eNOS/nitric oxide signaling pathway	(78)
LEC	limits lymphangiogenesis and reverse cholesterol transport	SPON2/LRG4/eNOS/ VEGFC/VEGFR3 signaling pathway	(79)
VSMCs	protects against vascular hyperplasia	AKT/GSK3β/mTOR/FOXO3A/FOXO1 signaling pathway	(80)

#### 4.2.1 Promotion of growth, development, and angiogenesis

SPON2 exerts a significant influence on the development of bone and muscle. Aoki M et al. have elucidated the critical role of SPON2 in maintaining the apical ectodermal ridge (AER) and its indispensability for growth and patterning during limb development (81). Hankenson KD et al. have reported that SPON2 facilitates osteoblast differentiation, while its deficiency results in skeletal developmental abnormalities (82). JinYR et al. revealed that SPON2 exerts a regulatory role in the morphogenesis of midfacial, limb, and lung structures during embryonic development, with this regulation being mediated via the WNT/β-catenin signaling pathway (17, 18). Wang H et al. discovered that SPON2 derived from prostate cancer (PRAD) cells significantly enhances the expression of osteogenic factors in osteoblasts through the PI3K/AKT/mTOR signaling pathway (69). Bell SM et al. identified a severe hypomorphic SPON2 allele that was associated with pulmonary abnormalities. Co-inheritance of the SPON2 (Tg) allele with the Lrp6(-) allele exacerbated these defects, resulting in pronounced lung hypoplasia and complete absence of tracheal-bronchial rings, laryngeal structures, and all limb skeletal elements (83). Furthermore, Kazanskaya O et al. revealed that depletion of SPON2 in Xenopus embryos failed muscle markers MYOD and MYF5 to activate, leading to impaired muscle development at a later stage (84). Becker D et al. identified a 50-kb deletion on chromosome 14 (Bos taurus BTA14) that disrupts the coding sequence of the SPON2 gene, thereby establishing an association between this deletion and bovine tetradysmelia (3).

Additionally, SPON2 plays a crucial role in the maintenance of tooth and hair follicle stem cells. Notably, Kawasaki M et al. have elucidated the involvement of the SPON2/LGR signaling pathway in tooth development (85). Arima M et al. identified SPON2 as a crucial regulator of osteoblastic differentiation in immature human periodontal ligament cells, specifically expressed in periodontal ligament tissue and cells, through the activation of the WNT/β-catenin signaling pathway (86). Smith AA et al. have demonstrated that SPON2 treatment induces activation of hair follicle stem cells, indicating its potential as a therapeutic agent for promoting hair growth (87).

SPON2 plays a pivotal role in both follicular development and angiogenesis, as demonstrated by Hwang SU et al., who highlighted the indispensability of SPON2 and the WNT/CTNNB1 signaling pathways in porcine follicle development (88). The study conducted by Cheng Y et al. has demonstrated the crucial role of oocyte-derived SPON2 as a paracrine factor in the development of primary follicles. These findings suggest that targeting SPON2 agonists could present a novel therapeutic approach for infertile women with diminished responses to conventional gonadotropin therapy (89). Termini CM et al. reported that systemic administration of anti-SPON2 effectively suppresses vascular regeneration and hematopoietic reconstitution. SPON2 exerts a promotive influence on vascular regeneration and hematopoietic reconstitution (90). Gerbaud P et al. reported that exogenous SPON2 promotes the proliferation of placental endothelial cells, while decreased secretion of SPON2 may impair placental vascular function in trisomy 21 syndrome (91).

#### 4.2.2 Promotion of cell proliferation

Chua AWC et al. unveiled the potential dual paracrine mechanism of keloid keratinocytes, whereby they induce upregulated expression of SPON2 in fibroblasts. This heightened SPON2 expression facilitates keratinocyte proliferation and epidermal thickening (92). Lin XL et al. propose that SPON2 may serve as a crucial neuronal factor responsible for maintaining taste tissue homeostasis through its modulation of taste stem cells (93). Gyllborg D et al. revealed the promotion of midbrain dopaminergic neurogenesis and midbrain dopaminergic neurogenesis in human embryonic stem cells by SPON2 (94). The regulation of this process by the WNT activator SPON2 was demonstrated by Hoekstra EJ et al. (95). Additionally, Yan H et al. revealed that SPON2 exerts a negative regulatory influence on oxidized low-density lipoprotein-induced macrophage apoptosis by modulating lipid uptake (96).

#### 4.2.3 Other biological functions

The SPON2 protein also plays a pivotal role in promoting inflammation, maintaining the integrity of the blood-gas barrier, and preserving homeostasis in tendons and ligaments. Zhang HY et al. observed that the polarization of synovial M1 macrophages exacerbates experimental collagenase-induced osteoarthritis, with SPON2 playing a partial role in this process. They propose that targeting both M1 macrophages and SPON2 could hold potential as therapeutic strategies for treating osteoarthritis (97). Li N et al. demonstrated the pivotal role of SPON2 in regulating macrophage migration and chemotaxis (98). Several scholars have identified SPON2 as a crucial determinant for maintaining the integrity of the blood-gas barrier (99). Zhu LH et al. demonstrated that SPON2 exerts regulatory control over hepatic lipid metabolism and effectively ameliorates hepatic steatosis, obesity, inflammation, and insulin resistance in mice (100). Tachibana N et al. observed that the expression of SPON2 was induced by both inflammatory stimulation and mechanical loading, acting through the nuclear factor κB pathway. They proposed that cells positive for SPON2 may have a role in maintaining tendon/ligament homeostasis, particularly under pathogenic conditions (101). Furthermore, Zhu C et al. demonstrated *in vivo* that the administration of exogenous SPON2 effectively mitigated bone loss and enhanced bone microstructure in OVX mice. SPON2 may function as a positive regulator of bone metabolism through the activation of the classical WNT/β-catenin signaling pathway (19).

Hepatic stellate cells, as non-parenchymal perihepatic cells, have garnered significant attention owing to their pivotal role in liver fibrosis. Yin XG et al. have identified that SPON2 may facilitate the activation of hepatic stellate cells by augmenting the canonical WNT pathway (102). The study conducted by Munguía-Reyes A et al. revealed an upregulation of SPON2 in Idiopathic Pulmonary Fibrosis (IPF), and notably, it appears to exert an antifibrotic effect within this context (103). The diverse roles of SPON2 in the pathogenesis of liver fibrosis and pulmonary fibrosis underscore its tissue-specific effects on fibrotic processes.

## 5 Clinical treatment strategy based on SPON2

Currently, SPON2 is being increasingly utilized in clinical diagnosis and treatment. The identification of SPON2 gene fusion, gene rearrangement, and SPON2 gene polymorphism offers valuable therapeutic insights for tumors.

Li C et al. investigated patient-derived xenograft (PDX) tumor RNA samples, identifying fusion events involving novel SPON2 transcribed genes and demonstrating the oncogenic role of SPON2-EMC2 fusion genes in tumorigenesis, tumor growth maintenance, and metastasis promotion. Subsequently, a WNT pathway inhibitor was employed to treat a PDX mouse model harboring the SPON2 fusion gene, resulting in a complete response and cessation of progression in all cases of SPON2 fusion tumors. These findings suggest that targeting the WNT pathway could serve as an effective therapeutic strategy for digestive system cancers characterized by SPON2 fusions, with the potential utility of SPON2 fusion as a biomarker for patient screening to support clinical implementation of WNT pathway inhibitors (104). Increasing evidence suggests that SPON2 gene rearrangement may serve as a key driver in the pathogenesis of CRC. Han T et al. developed an inducible CRISPR (iCRISPR) transgene platform to reprogram SPON2 expression in the mouse gut, providing direct evidence that endogenous EIF3E-SPON2 fusion events alone are sufficient to initiate intestinal tumor development (105). Ampulla adenocarcinoma is an infrequent malignant neoplasm, accounting for a mere 0.2% of gastrointestinal tumors. Linscott MP et al. have recently identified a novel SPON2 RNA fusion in a patient with recurrent metastatic ampulla adenocarcinoma. Remarkably, this patient achieved enduring remission of metastatic ampulla adenocarcinoma through the utilization of nanoparticle albumin-bound (nab) paclitaxel and gemcitabine combination chemotherapy. The authors propose that targeting the SPON2 RNA fusion could hold promise as a potential therapeutic strategy. Nevertheless, it is important to note that this study suffers from limitations due to its small sample size, necessitating further research to ascertain its applicability in treating similar patients (20).

Berger MD et al. conducted a study on 773 patients with metastatic colorectal cancer who received FOLFIRI/bevacizumab or FOLFIRI/cetuximab, aiming to assess the impact of six functional single nucleotide polymorphisms (SNPs) in Spondin-1, Spondin-2, and Spondin-3 genes on treatment outcomes. The findings indicate that the single nucleotide polymorphism rs555008 in SPON2 may serve as a predictive biomarker for identifying patients who can benefit from FOLFIRI/bevacizumab therapy in the context of metastatic colorectal cancer (21). The precise expression pattern of proteins in tumor cells serves as a crucial foundation for targeted therapeutic interventions. SPON2/RG-1, a homologous gene of the SPON2 protein, has been identified by Parry R et al. to exhibit selective expression within prostate tissue through comprehensive gene expression analysis. Based on these findings, the authors propose that the heightened expression levels of SPON2/RG-1 in prostate tumors render it a promising target for antibody-based radiotherapy (22).

Based on the aforementioned publicly available data, there have been promising preliminary findings in terms of clinical efficacy. Furthermore, we eagerly anticipate the outcomes of long-term studies or ongoing clinical trials investigating SPON2 in diverse tumor types, which may offer novel therapeutic options for patients, including those with colorectal cancer, ampulla adenocarcinoma, prostate cancer, and more.

## 6 Conclusions and perspectives

As a versatile biomarker, SPON2 expression is upregulated in various tumor types, providing valuable insights for the clinical diagnosis and treatment of over ten malignancies including prostate cancer and colorectal cancer. Moreover, alterations in SPON2 expression also hold significant potential implications for the diagnosis of certain non-tumor diseases. Functionally, SPON2 exhibits diverse roles; it can function as either an oncogene or a tumor suppressor gene depending on the specific tumor type, regulating tumor cell proliferation, invasion, and metastasis. In non-tumor tissues, it plays a pivotal role in follicle development, embryogenesis, limb formation, and midfacial morphogenesis. Furthermore, SPON2 participates in multiple signaling pathways with distinct biological functions. Notably, there have been notable advancements in developing clinical treatment strategies based on targeting SPON2.

Currently, numerous studies on SPON2 have contributed to a more comprehensive understanding of various diseases. However, future investigations should focus on refining the definition of the high-expression population for SPON2, predicting marker efficacy, implementing measures to prevent and control adverse reactions, selecting treatment plans for populations with multi-target co-expression, and integrating immunotherapy. These areas represent crucial directions for further exploration. Subsequent clinical trials will undoubtedly offer additional therapeutic options for patients exhibiting high SPON2 expression and poor drug response.

## Author contributions

JZ: Writing – original draft. GL: Writing – review & editing. YL: Writing – review & editing. PY: Writing – review & editing. JX: Writing – review & editing. XW: Writing – original draft, Writing – review & editing.
